# Predictors of Balloon Guide Catheter Assistance Success in Stent-retrieval Thrombectomy for an Anterior Circulation Acute Ischemic Stroke

**DOI:** 10.7759/cureus.5350

**Published:** 2019-08-08

**Authors:** David J McCarthy, Samir Sur, Adisson Fortunel, Brian Snelling, Evan Luther, Dileep Yavagal, Eric Peterson, Robert M Starke

**Affiliations:** 1 Neurosurgery, University of Miami Miller School of Medicine, Miami, USA; 2 Neurosurgery, Boca Raton Regional Hospital, Boca Raton, USA; 3 Neuroendovascular Surgery, University of Miami Miller School of Medicine, Miami, USA

**Keywords:** ischemia, large vessel occlusion, mechanical thrombectomy, outcomes, stroke, balloon guide, stent retriever

## Abstract

Introduction

Mechanical thrombectomy has become the standard treatment for large vessel occlusion (LVO) in acute ischemic stroke (AIS) in well-selected patients. Although many devices and strategies exist, the use of a balloon-tip guide catheter (BGC) with stent-retriever (SR) may hold several advantages. We aim to assess the efficacy and identify predictors of technical success of this unique approach.

Methods

From our prospectively maintained database, we identified consecutive cases in which a BGC was used for stent-retriever thrombectomy in anterior circulation LVO between 2015 and 2016. Baseline and procedural characteristics were captured and analyzed. Predictors of technical and clinical outcomes were identified by multivariable logistic regression analysis.

Results

Ninety-three patients with AIS-LVO were treated with BGC-assisted mechanical thrombectomy. The mean age was 71 years old (SD 14), with 49.5% male (n=46). Pre-operative IV-tPA was administered in 55.9% (n=52) of cases. The most common location of occlusive thrombus was M1 (64.5%, n=60). Successful recanalization (mTICI=2b-3) was achieved in 86.0% (n=80) of cases while complete revascularization (mTICI-3) was achieved in 56.5% (n=52). There was a first-pass success rate of 52.7% (n=49). At discharge, 38.7% of the patients were functionally independent (mRS≤2). Multivariate analysis revealed that the middle cerebral artery location was strongly predictive of first-pass success, resulting in mTICI =2b revascularization (OR 7.10, p=0.018). Additionally, female gender (OR 2.85, p=0.042) and decreasing mTICI were associated with a poor clinical outcome (mRS≥4; OR 1.76, p=0.008).

Conclusions

BGC assistance in stent retrieval thrombectomy is safe and effective for AIS due to anterior circulation LVO. Further investigation is required to elucidate the optimal treatment strategy based on patient and disease characteristics.

## Introduction

In 2015, five randomized prospective trials demonstrated a clear benefit of endovascular intervention for the treatment of acute ischemic stroke (AIS) of anterior circulation due to large vessel occlusion (LVO) [1-5]. Following the publication of these landmark randomized clinical trials, mechanical thrombectomy (MT) became the standard of care for AIS due to LVO. Currently, efforts have been directed towards optimizing patient outcomes through the evaluation of the multiple thrombectomy techniques [6].

Currently employed MT techniques include stent retriever (SR), with or without balloon-tip guide catheter (BGC), aspiration at the face of the clot (ADAPT), and combinations of direct aspiration at the thrombus with the simultaneous deployment of a stent retriever (Solumbra technique) [7-14]. Despite reports of success with each of these techniques, the optimal strategy based on patient and disease characteristics remains unknown. Specifically, the use of a balloon guide catheter in combination with stent retrieval has been widely described, however, its utility remains unclear [7,9,12]. Only two of the five 2015 RCTs recommended BGC usage, with only the REVASCAT (REVASCAT) study reporting the BGC-assistance rate (60%). Multiple retrospective analyses report that BGC-assisted thrombectomy results in shorter procedure times and improved revascularization compared to NBGC [8,10,15-16]. Regardless, stroke registries report that only 50% of thrombectomies are performed with BGC assistance and there are a number of potential advantages to non-balloon guide thrombectomy approaches [8].

We report our single-institution series of BGC-assisted SR. We hypothesize that our series will report the clinical and technical benefits of BGC assistance and demonstrate the necessity for a more adequately powered randomized investigation to determine the optimal approach. Additionally, we sought to identify specific patient and procedural factors associated with favorable outcomes following BGC assistance.

## Materials and methods

Patient selection

Following local institutional board approval, we reviewed our prospectively maintained database of AIS interventions, identifying consecutive cases of stent retrieval thrombectomy for anterior circulation LVO in AIS from February 2015 until September 2016 at Jackson Memorial Hospital (Miami, Florida). We included only anterior circulation BGC-assisted MT, excluding MT without BGC assistance and posterior circulation clots. A total of 93 patients who underwent stent retrieval thrombectomy for acute ischemic stroke met these criteria.

Upon arrival at the hospital emergency department, patients received rapid non-contrast computed tomography imaging (CT), CT-angiography, and examination by an on-call neurologist. If medically appropriate, patients were treated with IV-tPA prior to cerebrovascular intervention. Stable patients received midazolam and fentanyl for sedation, whereas intubation was required for patients unable to protect the airway or remain still for the procedure.

Endovascular technique

Femoral access was obtained and an 8F or 9F vascular sheath was placed. Preoperative analysis of the aortic arch on CT angiography was often used to select the intermediate catheters and guide wires. In general, an 0.035” guidewire was used to navigate a 125-cm diagnostic catheter into the ipsilateral carotid artery, and the BGC was then advanced over the diagnostic intermediate catheter and wire to achieve an optimal position in the mid or high cervical internal carotid.

Once the BGC was in place and LVO had been confirmed by angiography, a microcatheter was advanced into the selected vessel over a shaped microwire. Microangiography was often used to confirm the placement of the microcatheter distal to the thrombus and the stent retriever was subsequently deployed through the microcatheter across the thrombus. After five minutes elapsed, the balloon was inflated in the internal carotid artery (ICA) under fluoroscopy and the stent retriever was pulled, along with the microcatheter, through the BGC with simultaneous aspiration from the BGC.

Follow-up angiography was then performed through the BGC after the balloon was deflated. If thrombus remained, the microsystem was redeployed and another pass with the stent-retriever was attempted.

Outcomes and variables

The main endpoints analyzed were technical and clinical outcomes and complications. Recanalization was assessed using the modified Thrombolysis in Cerebral Infarction (mTICI) score; mTICI scores of 2b or 3 were deemed successful reperfusion while complete revascularization was defined as mTICI 3. Clinical outcomes were assessed using the modified Rankin Score (mRS), with favorable outcomes defined as mRS of 2 or less; unfavorable outcomes were defined as mRS 4 or more. Complications that were studied included hemorrhagic conversions seen on radiographic imaging, subsequent embolic events either during the procedure or same hospital stay and death.

To identify predictors of successful BGC-assisted thrombectomies, the following variables were analyzed: gender, age, time from ED to procedure, time from onset of stroke to procedure, thrombus location, tPA bolus administration, microcatheter intra-arterial (IA) tPA administration, procedural times, first-pass success (first attempt with thrombectomy device removed occlusion), and complications.

Statistical analysis

Data are presented as the mean and range for continuous variables and as the frequency for categorical variables. Bivariate comparisons between successful and unsuccessful reperfusion groups were made using the student t-test or Aspin-Welch-Satterthwaite t-test and χ2 test or Fisher's exact test, as appropriate. Independent predictors for success using regression analysis, carried out using the unpaired t-test, chi-square, Fisher’s exact tests, and Mantel Haenszel test for the linear association as appropriate. Univariable analysis was used to test covariates predictive of the following dependent variables: complete revascularization (mTICI=3), first-pass success resulting in revascularization (mTICI 2b, 2c, or 3), unfavorable outcome (mRS 4-6), and hemorrhagic conversion. Interaction and confounding were assessed through stratification and relevant expansion covariates. Factors predictive in univariable analysis (p<0.15) were entered in a multivariable logistic regression analysis. P-values of ≤0.05 were considered statistically significant. Statistical analysis was carried out with Stata 10.0 (College Station, TX, US) and S.A.S 9.4 (Cary, NC, US).

## Results

Between 2015 and 2016, a total of 93 patients with AIS due to LVO were treated with BGC-assisted stent retrieval thrombectomy. Cohort details are demonstrated in Table 1. The patients' mean age was 71 (SD 14), with 49.5% male (n=46). Pre-operative IV-tPA was administered in 55.9% (n=52) of cases. Average time from symptom onset until groin puncture was 316 minutes (IQR 131.5-382 min). Average intervention time, groin puncture to reperfusion, was 67.9 minutes (IQR 28- 83 min). The M1 segment was the most common location of occlusive thrombus (64.5%, n=60).

**Table 1:** Baseline characteristics, overall and by reperfusion success following BGC-assisted thrombectomy for stroke Values expressed as n (%) unless otherwise specified. Y indicated years; mTICI indicates modified treatment in cerebral ischemia score; IV-tPA indicates intravenous thrombolysis; NIHSS, National Institutes of Health Stroke Scale; min indicates minutes; MCA indicates middle cerebral artery; M1 indicated first MCA segment; M2, second MCA segment; M3, third MCA segment; ICA, internal carotid artery. *p-values calculated using the student t-test or Aspin-Welch-Satterthwaite t-test and χ2 test or Fisher's exact test as appropriate.

		Overall	Reperfusion success		P-value*
			No (mTICI<2b)	Yes (mTICI 2b,2c or 3)	
Number of patients		93	13 (13.0)	80 (86.0)	
Age, y; mean ± SD		71.1 ± 14.2	72.9 ± 17.6	70.8 ± 13.6	0.63
Male		46 (49.5)	3 (23.1)	37 (46.3)	0.07
Admission NIHSS; mean ± SD		16.5 ± 6.3	20 ± 4.4	16 ±6.4	0.016
IV-tPA bolus		52 (55.9)	4 (30.8)	48 (60)	0.049
General anesthesia		2 (2.2)	1 (7.7)	1 (1.25)	-
Onset to reperfusion time, min; median (IQR)		290 (289-475)	438 (260-975)	266.5 (173-425)	0.14
Groin puncture to reperfusion time, min; median(IQR)		51 (28-83)	101 (78-127)	43 (27-72)	0.009
Tandem ICA stenosis		7 (7.5)	1 (7.7)	6 (7.5)	-
Hemorrhagic conversion		25 (26.8)	6 (46.2)	19 (23.8)	0.18
Subsequent embolization		18 (19.4)	4 (30.8)	14 (17.5)	0.27
Occlusion location					
MCA		81 (87.1)	10 (76.9)	71 (88.8)	0.36
	M1	60 (64.5)	7 (53.9)	53 (66.3)
	M2	19 (20.4)	3 (23.1)	16 (20)
	M3	2 (2.2)	0 (0)	2 (2.5)
ICA		12 (12.9)	3 (23.1)	9 (11.3)	0.36

Procedure characteristics and outcomes

Successful recanalization of the LVO (mTICI ≥2b) was achieved in 86.0% (n=80) of cases, with complete revascularization of mTICI 3 in 56.5% (n=52). First-pass success rate was 52.7% (n=49). Machine aspiration assistance was used in 17 cases (18.3%). Intubation was required in 5 cases (5.4%).

Mean baseline NIHSS at presentation was 16 (SD6), with an average NIHSS of 13 (SD 9) following the intervention. Patients were severely impaired upon presentation (mRS<3) in 80.7%. At discharge, 38.7% of patients were functionally independent (mRS≤2). All patients had mRS score prior to discharge from hospital; mean follow-up was 42 days, with 52 patients (55%) lost to follow-up. Mortality was 23.6% (n=22). Hemorrhagic conversion was observed in the postoperative imaging of 25 patients (27.5%), only four of these were symptomatic (4.3%). Subsequent embolization to either vascular territory distal to the clot or novel territory occurred in 18 patients (19.4%).

Factors associated with radiographic or clinical outcome

Baseline characteristics and operative details were entered into a multivariate analysis to determine predictors of successful BGC-assisted stent retrieval thrombectomy, seen in Table 2. Isolated occlusions located in the middle cerebral artery (MCA) had a higher rate of complete revascularization, as well as first-pass success resulting in revascularization when compared to an alternative thrombus location. Patients who received preoperative IV-tPA bolus had a higher rate of first-pass success resulting in revascularization. Patients with tandem internal carotid artery (ICA) stenosis were less likely to have a successful first pass (tandem first pass n=1, 14.3%; tandem failed first pass n=6, 85.7%; OR=8.55; p=0.056).

**Table 2:** Multivariate logistic regression analysis of factors associated with BGC-assisted stent retrieval thrombectomy MCA indicates middle cerebral artery; IV-tPA, intravenous tissue plasminogen activator; ICA, internal carotid artery; mTICI, modified thrombolysis in cerebral infarction; OR, odds ratio; CI, confidence interval.

Factors associated with success	OR (95% CI)	p-value
Complete revascularization (mTICI=3)		
M1 MCA thrombus	3.4 (1.36-8.50)	0.009
Interarterial-tPA	0.43 (0.17-1.04)	0.062
First pass success		
Preoperative IV-tPA bolus	2.88 (1.21-6.87)	0.017
ICA tandem stenosis	0.117 (0.01-1.05)	0.056
First pass success resulting in revascularization (2b ≥ mTICI)		
MCA thrombus	7.1 (1.39-36.1)	0.018
Preoperative IV-tPA bolus	3.28 (1.34-8.03)	0.009
Hemorrhagic conversion		
Interarterial-tPA	4.11 (0.08-0.79)	0.018
Unfavorable outcome at last interaction (mRS 4-6)		
Decreasing mTICI	1.76 (1.15-7.83)	0.008
Female gender	2.85 (1.04-7.83)	0.042
Hemorrhagic conversion	8.33 (2.41-28.79)	0.001
Puncture to perfusion time	1.01 (0.99-1.03)	0.07

Significant multivariate predictors for unfavorable outcome included decreasing mTICI score, female gender, and hemorrhagic conversion as seen on postoperative CT scan (Table 2). Use of intraoperative tPA delivered arterially through a microcatheter was associated with postoperative hemorrhagic conversion as well as a lower complete revascularization rate.

## Discussion

Our single-institution prospective study investigated 93 patients with anterior circulation LVO AIS-treated BGC-assisted stent retrieval thrombectomy. The technical and clinical outcomes of our series were similar to the reported rates of recanalization, high first-pass success, and favorable clinical outcomes [8,10]. At discharge, 38.7% of patients were functionally independent (mRS≤2). Identified predictors of BGC-assisted stent retrieval success included MCA thrombus location, preoperative IV-tPA bolus, and absent ICA tandem stenosis. Low mTICI score, female gender, and hemorrhagic conversion were negative predictors of functional outcome.

In our cohort, MCA occlusion location was the greatest predictor of BGC-stent retrieval first pass success achieving revascularization. Other studies report MCA occlusion location as a positive prognostic indicator. The 2012 prospective 50 patient study, “Prognostic factors related to clinical outcome following thrombectomy in ischemic stroke (RECOST study)” reported that the MCA location was a positive predictor for recanalization for BGC-stent thrombectomy (70% in MCA vs 43% in ICA, p<0.04) [17]. Although the RECOST study primarily investigated outcomes and safety of stent retrieval thrombectomy, the investigators recognized the benefits of BGC-assistance and included it in their protocol. Additionally, Blanc et al. found that MCA location was predictive of successful revascularization for the aspiration component in the ADAPT technique (OR 2.48, CI 1.59-3.86, p<0.001). This may be the case with the ADAPT approach because the smaller clots that tend to occlude the MCA are easier to navigate to and form an ideal clot to catheter diameter surface, leading to better aspiration [18].

Furthermore, preoperative medical treatment with IV-tPA was associated with higher complete revascularization as well as first-pass success; however, patients without IV-tPA medical treatment were likely beyond the five-hour treatment window, which could inherently make successful first pass and revascularization more difficult to obtain. There was a strong trend for ICA-tandem stenosis to disrupt first-pass success. This is likely due to the complexity of pathology in these patients, often combining tortuosity and carotid bifurcation pseudo-occlusions with additional distal MCA occlusions.

While investigating aspiration in ADAPT, Blanc et al. also found that shorter onset to intervention time resulted in better recanalization, an observation we failed to see in our BGC-assisted stent retrieval cohort [18]. In our series, age and gender had no correlation with revascularization success; however, female gender was predictive of an unfavorable clinical outcome. Some reported literature has suggested that female gender is a negative prognostic factor for clinical outcomes following both thrombectomy and medical management for stroke [19-20].

Though limited by retrospective scope, several investigations of BGC-assisted thrombectomy vs. non-BGC thrombectomy report that BGC-assistance results in superior recanalization rates, shorter procedure times, higher first-pass success, and better 90-day clinical outcomes [8,10,15-16]. Brinjikji et al. performed a meta-analysis of the literature showing that patients treated with BGC had higher mTICI 3 (OR 2.13, 95% CI 1.43 to 3.17), mRS 0-2 (OR 1.84, 95% CI 1.52 to 2.22), and lower odds of mortality (OR 0.52, 95% CI 0.37 to 0.73) when compared with non-BGC patients.

Primary benefits of BGC-assisted thrombectomy stem from flow reversal during clot retrieval and aspiration, reducing clot fragmentation, distal embolization, and improving chances of clot retrieval [21-25]. Clinically, Lee et al. and Oh et al. found that BGC assistance resulted in significantly less distal embolization when compared to non-balloon guide catheter (NBGC) thrombectomy (OR, 6.3; 95% CI, 2.2-18.0; p<0.001) and (23.1% vs. 57.1%, p=0.02) [25-26]. In vitro investigation also found that BGC assistance resulted in better recanalization rates with less distal embolization (p<0.01) while suggesting that the benefits of BGC assistance may extend beyond detectable clinical and radiographic findings due to microembolic fragments [21,27]. While the previously mentioned clinical studies defined distal embolization as new emboli to the distal or new vascular territory as observed on angiography, future analysis should consider utilizing MRI to compare post-BGC vs. non-BCG reperfusion in TICI 3 cases.

More recently, Maegerlein et al. investigated BGC-assisted stent retrieval with direct thrombus aspiration or BGC-assisted Solumbra. They called this new technique PROTECT [28]. Comparing PROTECT to the traditional Solumbra technique, they found that PROTECT had shorter procedure time (29 vs 40 min, p=0.002) as well as superior complete revascularization rates (70% vs 39%; p<0.001).

Beyond the benefits seen with regards to proximal flow arrest and decreased emboli, BGCs offer several technical advantages. They may require less maneuvering than distal aspiration catheters and simplify navigation through tortuous vessels while increasing proximal support [29]. Modern BGCs allow for intermediate catheter placement through the balloon guide. The limitations of BGC catheters include a smaller inner to outer lumen ratio and decreased trackability through tortuous anatomy as compared to standard support catheters. This may preclude access in tortuous patients or decrease the distal distance of access. Critics of BGC implementation argue that balloon preparation increases time to reperfusion, however; we avoided this by prepping the balloon during time allotted for stent-clot integration. Theoretically, BGCs do contain a risk of injury to the internal carotid artery (ICA) during balloon inflation; however, our cohort had zero incidences of vessel injury. Furthermore, comparative studies found no difference in vessel dissection or perforation between BGC and non-BGC techniques [8,10,25]. A large pool of retrospective literature reports substantial benefits seen with BGC assistance; however, the results haven’t been translated into practice due to the lack of evidence from an adequately powered randomized clinical trial.

Our study has limitations including the outcomes of a single-center experience, which leads to selection bias. The small sample size limited the study power. As such a number of variables might be predictive of the outcome but were not found to be significant due to type II error. Furthermore, long-term clinical outcomes are necessary.

## Conclusions

The use of a BGC in stent retrieval thrombectomy results in a high rate of technical success and excellent clinical outcomes in anterior circulation LVOs. While the optimal strategy for performing thrombectomy remains unclear, our data suggest that the middle cerebral artery occlusion location predicts BGC-assisted stent retrieval success. While BGC assistance offers operator maneuverability with support, there is no substantial evidence that it is the most beneficial technique for the patient. Further investigation is required to elucidate the optimal treatment strategy based on patient and disease characteristics. An adequately powered randomized clinical trial is indicated.
